# Permanent magnet actuation for magnetic bead-based DNA extraction

**DOI:** 10.1186/s12938-018-0572-7

**Published:** 2018-11-06

**Authors:** Chang-Young Park, Young-Hyun Park, Yu-Seop Kim, Hye-Jeong Song, Jong-Dae Kim

**Affiliations:** 1 Department of Convergence Software, Hallym University, Chuncheon, South Korea; 2 Bio-IT Research Center, Hallym University, Chuncheon, South Korea

**Keywords:** DNA extraction, Magnetic bead, Permanent magnet, Solenoid actuator, Solenoid coil

## Abstract

**Background:**

Recently, automatic molecular diagnostic devices to extract DNA have been extensively developed using magnetic beads. While various methods can be applied to the control of the beads, the efficiency of the control when incorporated in automatic devices has not been studied. This paper proposes a compact magnet actuation method for the control of magnetic beads for DNA extraction, and compares the efficiency to the already available magnetic bead-based DNA extraction device. A permanent magnet was preferred for its compactness, while an electro-magnet provides easy operation. After investigating various methods to actuate the magnet with perspective to the size, circuit complexity, and power requirement, we determined the solenoid actuation method to be most efficient. To further reduce the dimension of the overall actuation device, direct actuation of the permanent magnet to control the hold/release of the beads was employed in this paper. The proposed method was compared with the conventional solenoid actuator with a metal plunger. An experimental fluidics device was set up with a fluidic channel and a syringe pump. The bead holding performance against the fluid speed was tested while a fixed amount of beads was loaded into the center of the channel. The group velocity of the beads was analyzed via image processing to determine whether the magnet was sufficient to hold the beads. The required power and space was analyzed and compared qualitatively and quantitatively.

**Result:**

The proposed direct actuation method was capable of holding the beads at faster fluidic speed than the conventional solenoid actuator. The required power was comparable contemplating the high initial power of the solenoid actuator, and required much smaller space since no plunger was needed.

**Conclusions:**

The direct actuation of the permanent magnet using a solenoid coil showed enhanced performance in holding the beads via permanent magnet, with less complexity of the actuation circuit and space. The proposed method therefore can efficiently improve the overall performance of the bead-based DNA extraction.

## Background

Molecular diagnostics is widely adapted in various fields such as disease detection and health monitoring. This method evaluates the nucleic acids (e.g., DNA, RNA, or a variation of both) for human samples as well as bacteria or virus which are the causes of many diseases [1–6]. The process examines the nucleic acids to determine the status of diseases and investigate the agent responsible for the infections. Molecular diagnostics follows four basic steps of sample collection, gene extraction from the collected sample, gene amplification by polymerase chain reaction (PCR), and analysis. The gene amplification step enables the diagnosis to be extremely accurate with high sensitivity and specificity.

The gene extraction from the sample is one of the most critical steps in the vast majority of recently developed automated DNA analysis devices [4, 7–14]. Accordingly, various studies have focused on methods to improve the efficiency of gene extraction, including the magnetic-bead based DNA extraction [3, 7, 8, 15]. Many automatic equipments for DNA analysis purpose adopted this technique due to its advantages of automation and application. Magnetic beads are widely used not only in DNA analysis, but also in diverse biochemical analysis using fluidics owing to the facile control of magnet beads with a magnetic force [4, 10, 12, 16–20].

In most researches, a permanent magnet is placed in close proximity to the region of interest in the microfluidic pathway to generate magnetic force to control the magnet beads [3, 16]. For the magnetic bead based extraction to be employed in automated devices, an electromagnet or a permanent magnet with an actuator is required to enable the binary operation of hold/release of the beads. Following the interest of end users that requests biochemical analysis equipments to be more compact and portable, we determined that a permanent magnet to be more suitable in improving the devices. An electromagnet is disadvantageous in regards to dimension since it becomes larger to produce the magnetic force comparable to a permanent magnet. By placing the permanent magnet in proximity to the beads by utilizing a motor or a solenoid actuator will efficiently decrease the size of the device. Although servo or stepper motors can be considered as an alternative, it has no advantage over a solenoid actuator with respect to the system complexity and the required space. For motors to be employed in a magnetic bead based extraction equipment, it requires an additional step for setting the home position upon assembly, and the control software of a stepper motor is also relatively complicated, when only the binary operation such as the hold/release of magnetic beads is required. Hence, this study focuses on the solenoid actuation methods for compact and portable analysis equipments.

While commercial solenoid actuators embed metal plungers, a permanent magnet can provide more advantages such as a relatively larger magnetic force and faster response [21, 22]. This paper proposes a direct actuation of the permanent magnet using a solenoid coil without the need of a metal plunger. Since the permanent magnet will be the plunger of the solenoid actuator, this method will reduce the space required to a great extent. However, the performance of the permanent magnet actuation via solenoid coil needs to be determined since the interaction between the permanent magnet and exposed magnetic force of the solenoid coil might effect the generated magnetic field that controls the magnetic beads.

The solenoid actuator with a metal plunger (solenoid actuator from hereafter) generates the largest force when the metal plunger is completely inserted [23]. Therefore, the power consumption can be minimized by inserting the metal plunger completely when holding the beads and removing it completely for release. This can be realized with a push-type solenoid actuator where the metal plunger is out of the solenoid coil using a spring in the release position. However, this type of solenoid actuator requires initial high current when actuated to the hold position due to the low force generated when the plunger is out of the solenoid coil. Consequently, a two-step circuit that can lower the initial current and prevent the solenoid actuator from being heated when the plunger is inserted to reach the hold position is required. In contrast, if a permanent magnet is driven directly with a solenoid coil, this two-step circuit is not required and can be implemented with a simple switch.

The distribution of the magnetic field can be analyzed through simulation or measurement to investigate the interaction of the permanent magnet and the solenoid coil [21, 24]. This study focuses on comparing the bead-holding performances of the two methods through a fluidic channel emulator [24]. The bead movement according to the fluidic velocity is analyzed using image processing to determine to what speed the magnetic force can efficiently hold the beads. We also performed a visual inspection of the bead movement to verify the image processing results. The experimental results indicate that directly actuating a permanent magnet with a solenoid coil is more advantageous over a solenoid actuator.

## Methods

We emulated a fluidic channel by creating a 60 mm by 5 mm channel on silicon rubber with the thickness of 0.8 mm (Fig. 1a). An acrylic sheet was used as the bottom and top cover of the silicon channel, and an inlet and outlet are placed on the top cover. As shown in Fig. 1b, two aluminum plates were placed and pressed down on the outer side of the acrylic covers to prevent leaking. The inlet and the outlet with 3 mm internal diameters were connected to a home-made syringe pump and a waste basket with silicon tubes (Fig. 2). The syringe pump is consisted of a 50 ml syringe, a commercial linear stage (MOX-02-30, Optics Focus Instruments Co., Ltd., China), and a commercial motor driver (MBCD-13A, Motion Bank, Korea).

**Fig. 1:** Fluidic emulator

**Fig. 2:** Fluidic emulator setup

The beads and permanent magnet used in this study were obtained from a commercial DNA extraction kits (MagAttract Suspension G, Qiagen, Germany). The procedure was repeated for various fluidic speeds. Since this study aimed to assess the bead-holding performances when the permanent magnet was actuated by the solenoid actuator to that of an independent solenoid coil, the solenoid coil used in the proposed method was obtained by disassembling the control subject (i.e., solenoid actuator, M060160H, Shindengen, Japan). The experiment procedure was as follows: loading the 9 μl bead solution at the channel center while the silicon channel is placed on the acrylic base; assembling the cover and the aluminum plates; and recording the bead movement using an industrial video camera (Chameleon, Point Grey Research, Inc., USA) while pumping the fluids with the syringe at a given velocity.

Figure 3 shows the two comparative subjects, the solenoid actuator and the solenoid coil placed together at the same distance to that of the fluidic emulator. The permanent magnet made of neodymium with the diameter of 8 mm and height of 15 mm is displayed above the metal plunger placed at the relative location when it is raised to hold the beads. It should be noted that in the actual experiment, only one of either the solenoid actuator or the solenoid coil is arranged in the center. The operation in the solenoid actuator experiment was performed by fixing the permanent magnet on top of the metal plunger. The movement of the permanent magnet was limited in vertical orientation using an acrylic cylinder.

**Fig. 3:** Metal-plunger solenoid actuator and its solenoid coil

The initial release position was determined to be 10 mm away from the acrylic base of the fluidic emulator, which is twice as far from the distance where the fluidic emulator showed no influence on the magnetic beads at the fluid speed of 100 mm/s.

The fluid velocity was calculated by dividing the volume speed by the cross-section (0.8 mm × 5 mm), in which the volume speed was calculated by measuring the time to release the entire 20 ml from the syringe under assuming laminar flow condition. A video camera was installed above the fluidic emulator to film the movement of the beads, and each frame was analyzed to observe the bead movement according to the fluid velocity. An image processing toolbox software based on MATLAB was utilized to measure the change in the bead group position (Fig. 4). The original images of the beads before and after the movement (left column of Fig. 4) were changed to a gray level and threshold with a fixed threshold to deliver binary images (middle column of Fig. 4). We attached a white paper on the bottom surface of the fluidic emulator and adjusted the lighting to enable efficient separation the beads to the background with the fixed threshold. The binary images were filtered by applying each of the morphological opening and closing with a 1-pixel radius (last column of Fig. 4). The holding performance was investigated by tracking the centroid of the white objects in the processed images according to time. The fluidic velocities from 100 to 1000 mm/s were tested and the velocities where the bead began to move were identified. The beads began to move between 500 and 600 mm/s for both methods, therefore experiments for those velocities were performed with precision.

**Fig. 4:** Imaging process used to measure the bead movement according to fluid velocity (from the left: original images, thresholded binaries, and morphologically filtered binaries)

## Result

The consumption power of the solenoid actuator and the solenoid coil to maintain the magnet at the hold position (10 mm from the actuators) was measured, and the solenoid coil consumed more power by 25%, with 144 mW and 180 mW for the solenoid actuator and the solenoid coil, respectively. However, taking into consideration that the solenoid actuator was twice as long, the power consumption of the solenoid coil is comparable to the actuator with twice more windings of coil. In electromagnet theory, the magnetic field and force generated by a solenoid is correlative to the length and number of windings a solenoid has. Therefore the power required for the solenoid coil to maintain the holding distance can be further reduced by increasing the winding of the coil.

The linear relationship between the motor jogging speed and the fluidic velocity was investigated to ensure that the acceleration of the motor drive did not influence the velocity of the fluid. The coefficient of determination (R2) of 0.9975 was obtained verifying the linearity of the motor jogging speed and fluid velocity, and that the number of the missing steps and the accelerating time of the stepper motor could be ignored.

Figure 5 shows the changes in the bead group position according to fluid velocity obtained by image processing. The top and bottom graph illustrates the result of the solenoid coil and solenoid actuator, respectively. Significant movement of beads were observed at 618 mm/s (top graph) and 580 mm/s (bottom graph) for the solenoid coil and actuator, respectively. This indicates that the solenoid coil paired with a permanent magnet had higher efficiency in holding the beads. Any change of the centroid location under 10 pixels over 100 frames was determined to be insignificant. A counterintuitive result was obtained in the case of the solenoid actuator where the bead movement was higher at 502 mm/s than at 541 mm/s (bottom graph Fig. 5). Visual inspection confirmed that this discrepancy was caused by the initial shape of the beads when loaded on the emulated fluidic chamber (Fig. 6). Due to the dune shape of the beads loaded in the experiment for 502 mm/s in the solenoid actuator, the calculated location of the centroid was affected when the bead returned to a circular shape over time.

**Fig. 5:** Change in the bead group position according to time

**Fig. 6:** Change in the bead distribution at low fluid velocity

## Discussion

In this study, we discovered that directly actuating a permanent magnet with a solenoid coil was more efficient in holding magnetic beads in position than the conventional solenoid actuator. The magnetic force generated by the solenoid coil seemed to bring a synergistic effect with the magnetic force of the permanent magnet. In contrast, the solenoid actuator lost its performance efficiency due to the housing of the metal plunger that interrupted the magnetic force generated by the coil.

To confirm that the electromagnet needs more space as stated in the instruction, the bead holding performance of the electromagnet tested by locating the solenoid coil at the bottom of fluidic emulator and driving it with the allowed maximum power (4 W). But it could not hold the bead even at the velocity of 100 mm/s.

The proposed method in this study will aid significantly in the improvement of not only the magnetic bead based DNA extraction devices, but also any magnetic bead based microfluidic devices, by simplifying and reducing the size of the equipment as well as reducing the cost since it does not require a solenoid actuator. The image processing analysis employed in our study can also be applied to any bead-based biochemical application.

## Conclusions

This study qualitatively and quantitatively compared the permanent magnet-driving methods used to extract DNA using magnetic beads. We compared the existing method of using a metal plunger paired with a solenoid coil and the proposed method of directly actuating the magnet with a solenoid coil through image processing. The experimental results showed that the solenoid coil had higher performance in holding the magnetic beads in position compared to the solenoid actuator. From our study, it can be concluded that the actuation of the magnet using a solenoid coil is advantageous in terms of the complexity of actuation circuits, required space, and holding performance than the conventional solenoid actuator.
